# Research Progress of PI3K/PTEN/AKT Signaling Pathway Associated with Renal Cell Carcinoma

This article has been retracted.

**DOI:** 10.1155/2022/1195875

**Published:** 2022-08-21

**Authors:** Yakun Fang, Wenjun Ji, Chao Yan

**Affiliations:** ^1^Department of Obstetrics, Qingdao Municipal Hospital, Qingdao 266000, China; ^2^Department of Radiation Oncology, Qilu Hospital (Qingdao), Cheeloo College of Medicine, Shandong University, Qingdao 266035, China

## Abstract

Renal cell carcinoma is a common renal malignancy of the urinary system and the most malignant type of kidney cancer. Phosphatidylinositol 3-kinase (PI3K) is an intracellular phosphatidylinositol kinase associated with oncogene products such as v-src and with serine/threonine kinase activity, and its increased activity correlates with the development of several cancers. Protein kinase B (AKT) is a cyclic guanosine phosphate-dependent protein kinase that plays an important role in cell survival and apoptosis. Phosphatase and tensin homolog (PTEN), a newly discovered oncogene in recent years, participates in tumorigenesis and development by competing with tyrosine kinases for common substrates. The product encoded by PTEN was found to negatively regulate the PI3K/Akt signaling pathway, thereby inhibiting cell proliferation and promoting apoptosis. The PI3K/PTEN/AKT signaling pathway has also been identified in several studies as being involved in the development of several malignancies, including renal cell carcinoma. Radiotherapy is currently one of the most effective means of treatment for renal cell carcinoma, whereas it is predisposed to significant tolerance during the course of radiotherapy, thereby leading to treatment failure. Therefore, new treatment options may potentiate the efficiency of renal cell carcinoma treatment. With the development of tumor molecular biology, targeted biological therapy for malignant tumors has gradually become a research hotspot. Given the above research background, this study reviews the application of the PI3K/PTEN/AKT signaling pathway in renal cell carcinoma, aiming to provide more references for the treatment of clinical renal cell carcinoma.

## 1. Introduction

Renal malignancies are malignant tumors originating from the urinary tubular epithelium of the renal parenchyma, of which renal cell carcinoma accounts for about 90% [1]. A study on the incidence, prevalence, mortality, and survival of kidney cancer worldwide in the past decade found a rising stage of global renal cell morbidity and mortality [2]. In China, the incidence of renal cell carcinoma is second only to bladder cancer [3]. Currently, radiotherapy, chemotherapy, and surgery are the mainstays for the treatment of renal cell carcinoma, among which surgery is the most effective method. Nevertheless, patients with advanced or metastatic disease are predisposed to recurrence and metastasis after surgery [4]. Chemotherapy has cytotoxic and differentiation-promoting effects which inhibit the growth of tumor cells and promotes their differentiation, but it simultaneously kills tumor cells and damages normal cells. Moreover, renal cell carcinoma has been reported to be significantly tolerant to chemotherapeutic agents [5]. Due to the presence of radiation resistance, some patients with renal cell carcinoma treated with radiotherapy may develop recurrence and metastasis [6]. Targeted therapy is a treatment modality that specifically selects cancer-causing sites at the cellular molecular level by designing corresponding therapeutic drugs for the identified cancer-causing sites, resulting in the specific death of tumor cells without affecting normal cells. However, issues such as drug resistance and adverse reactions give rise to the failure of long-term remission in some patients with renal cell carcinoma after targeted therapy [7]. Therefore, the exploration of new therapeutic targets has captured great attention in renal cell carcinoma research at this stage. A recent study has revealed that the activation of the PI3K/PTEN/AKT signaling pathway inhibits the induction of apoptosis in tumor cells by exogenous stimuli, which consequently promotes cell proliferation and metastasis [8]. Moreover, it has been suggested that blocking the activation of its effector molecules by inhibiting the PI3K/PTEN/AKT signaling pathway could potentially serve as a new idea for the treatment of renal cell carcinoma [9]. Accordingly, this study reviews the progress of PI3K/PTEN/AKT signaling pathway research in renal cell carcinoma.

## 2. PI3K/PTEN/AKT Signaling Pathway Components

Phosphatidylinositol 3-kinase (PI3K) is an intracellular phosphatidylinositol kinase consisting of a regulatory subunit and a catalytic subunit. PI3K is commonly divided into 3 categories according to differences in structure and function, among which PI3K-*α* is the most widely studied. PI3K can be initiated by various growth factors or signaling complexes such as vascular endothelial growth factor and fibroblast growth factor, which consequently regulate various cellular functions such as cell proliferation, differentiation, and apoptosis [10]. The PI3K/AKT signaling pathway plays a key regulatory role in the development of multiple malignancies [11]. Phosphatase and tensin homolog (PTEN) is the first oncogene with bispecific phosphatase activity identified to date and is another gene closely related to tumorigenesis after the P53 gene, with prime roles in cell growth, apoptosis, adhesion, migration, and infiltration [12]. Previous study has confirmed the involvement of the PI3K/PTEN/AKT signaling pathway in the pathogenesis of various malignancies [13]. Therefore, therapeutic strategies targeting the PI3K/PTEN/AKT signaling pathway may provide new ideas for tumor treatment.

## 3. The Relationship between PI3K/PTEN/AKT Signaling Pathway Activation and Renal Cell Carcinoma

It has been found that the activation of the PI3K/AKT signaling pathway promotes epithelial-mesenchymal transition and invasion of renal cancer cells and participates in the malignant transformation of renal cancer cells [14]. As kidney cancer cells express more drug-resistant proteins, they are less responsive to immunotherapy, chemotherapy, and radiotherapy [15]. It has been reported that the overactivated PI3K/AKT signaling pathway is one of the main causes of multidrug resistance in tumor cells [16]; therefore, targeting or blocking the expression of the PI3K/Akt signaling pathway may potentially reverse drug resistance in tumor cells. Long et al. [17] revealed a significant downregulation of PTEN expression in renal cell carcinoma, which correlates remarkably with clinical stage, histological grade, lymph node, and distant metastasis. Moreover, another study also indicated that deletion and abnormal expression of PTEN may be associated with renal cell carcinogenesis [18]. Recent research has revealed that inactivation of PTEN may lead to abnormal activation of the PI3K/AKT signaling pathway and promote tumor cell growth, invasion, and metastasis [19].

The PI3K/AKT/PTEN signaling pathway serves as a potential molecular target to control tumorigenesis by regulating cell division, tumor growth, angiogenesis, apoptosis, invasion, and cellular metabolism in tumor and stromal compartments [20]. Furthermore, activation of the PI3K/PTEN/AKT pathway has been associated with malignant pathogenesis and the development of drug resistance [21]. Zheng et al. [22] found that interference with PI3K/AKT/PTEN signaling significantly ameliorated tacrolimus-induced kidney injury. Xiaoli et al. [8] inhibited PI3K/PTEN/AKT pathway signaling by silencing the TP53 gene, which markedly inhibited PTEN-induced infiltration and metastasis of renal clear cell carcinoma.

## 4. PI3K/PTEN/AKT Signaling Pathway and Multidrug Resistance in Renal Cell Carcinoma

Multidrug resistance in kidney cancer is considered the main factor leading to unsatisfactory chemotherapy results or even failure of treatment in kidney cancer patients [23], and multiple drug-resistant genes present in kidney cancer are predisposed to resistance to a single targeted agent, which substantially compromises the efficacy [24]. Accordingly, a consensus has been developed among some scholars that the combination of drugs with different targets may potentiate therapeutic efficiency. Previous investigation has shown that the PI3K/Akt signaling pathway is a potential target for chemotherapy resistance treatment, and inhibition of its signaling may effectively diminish the occurrence of drug resistance [25]. It has been demonstrated that overexpression of PTEN significantly inhibits the proliferation of esophageal cancer cisplatin-resistant cell line Ec9706/cDDP cells, promotes their apoptosis, and reduces the expression of P-glycoprotein, a key tumor resistance protein, thereby reversing multidrug resistance in esophageal cancer cells [26]. Another study indicated that the sensitivity of kidney cancer cells to sunitinib is mediated by the regulation of the expression of the oncogene PTEN, which may allow sunitinib to exert its inhibitory effect on kidney cancer cell activity at lower concentrations [27]. The above findings suggest that homoregulation of the PI3K/PTEN/AKT signaling pathway may be valuable for the reversal of multidrug resistance in renal cell carcinoma.

## 5. Targeting PI3K/PTEN/AKT Signaling Pathway Molecules in the Treatment of Renal Cell Carcinoma

The use of targeted therapies has improved clinical outcomes in patients with metastatic renal cell carcinoma; however, resistance to targeted therapies may develop in most patients over time, which compromises therapeutic efficacy [28]. Therefore, the quest for new targets for intervention bears great significance in improving the prognosis of patients with renal cell carcinoma.

### 5.1. PI3K Inhibitor

LY294002 is the first synthetic PI3K inhibitor that permeabilizes cells and specifically inhibits the expression of PI3K-*α*, *β*, and *δ*, which consequently regulates the PI3K/AKT signaling pathway. It was shown that LY294002 promotes glycyrrhiza chalcone A-induced autophagy in kidney cancer cells [29]. Besides, blocking the AKT pathway with the specific inhibitor LY294002 reverses matrix metalloproteinase expression and negatively regulates renal cancer cell migration and invasion [30].

### 5.2. AKT Inhibitor

MK2206 is a potent, highly specific, non-ATP-competitive binding AKT inhibitor, with high inhibitory effects on AKT1 and AKT2 activity but little on AKT3 [31]. Akt inhibitor MK-2206 has been reported to regulate cancer cell biological behavior by modulating the PI3K/Akt signaling pathway [32]. A potential synergistic effect of MK2206 on enhancing radiotherapy sensitivity in patients with malignant tumors has also been revealed in a prior study [33]. Miransertib is a novel orally bioactive and selective AKT inhibitor with a favorable and modifiable safety profile in advanced solid tumors [34], but it has not yet been reported for the treatment of renal cancer. To the best of our knowledge, ARQ751 is also a potent and selective AKT inhibitor. At the American Society of Hematology 2019, ArQule presented data from the phase I clinical trial of ARQ751 showing that ARQ751 may be effective for the treatment of solid tumors carrying PKD3CA/AKT/PTEN mutations.

### 5.3. PTEN Agonists

PTEN is considered a dormant tumor suppressor gene. One study analyzed the correlation of PTEN with clinical stage, pathological type, foreman grading, overall survival, progression-free survival, and disease-specific survival in renal cancer and revealed a significant association of PTEN expression with unfavorable decision support systems. Specifically, its low expression may predict poor outcomes [35]. The proliferation and colony formation of kidney cancer cells were substantially inhibited by upregulation of PTEN expression, which induced cells to enter G1 phase arrest [36]. Nonetheless, no targeted drugs that directly agonize PTEN have yet been discovered. Ribosomal protein S6 kinase 1 (S6 kinase 1, S6K1) is an important substrate for mTOR. It was found that novel inhibitor molecules targeting S6K1 exert specific cytotoxic effects on PTEN-deficient cancer cells [37].

## 6. Prospects

The activation of the PI3K/PTEN/AKT signaling pathway for various causes promotes tumor progression and metastasis, which plays an important role in the genesis and development of many malignancies and has become a new target for tumor therapy [38]. However, the biological properties and mechanisms of action of this pathway have not been fully elucidated at home and abroad. In particular, in renal cell carcinoma, only one case has been reported [8, 39] on the relationship between PI3K/PTEN/AKT signaling pathway and renal cell carcinoma. Nevertheless, many issues remain. In addition, the role of PI3K/PTEN/AKT pathway target proteins in renal cell carcinoma is still poorly understood. Many of the new PI3K inhibitors, AKT inhibitors, and PTEN agonists are still in clinical trials, with unknown effects in renal cell carcinoma. The combination of three targeted drugs is expected to be a hotspot for future research in renal cell carcinoma. As research progresses, the PI3K/PTEN/AKT pathway is expected to become a more precise target to maximize the clinical efficiency of patients with renal cell carcinoma.

## Data Availability

All data was within the manuscript.
